# RLMD-PA: A Reinforcement Learning-Based Myocarditis Diagnosis Combined with a Population-Based Algorithm for Pretraining Weights

**DOI:** 10.1155/2022/8733632

**Published:** 2022-06-30

**Authors:** Seyed Vahid Moravvej, Roohallah Alizadehsani, Sadia Khanam, Zahra Sobhaninia, Afshin Shoeibi, Fahime Khozeimeh, Zahra Alizadeh Sani, Ru-San Tan, Abbas Khosravi, Saeid Nahavandi, Nahrizul Adib Kadri, Muhammad Mokhzaini Azizan, N. Arunkumar, U. Rajendra Acharya

**Affiliations:** ^1^Department of Electrical and Computer Engineering, Isfahan University of Technology, Isfahan, Iran; ^2^Department of Electrical and Computer Engineering, University of Kashan, Kashan, Iran; ^3^Institute for Intelligent Systems Research and Innovation (IISRI), Deakin University, Waurn Ponds, Victoria 3216, Australia; ^4^Dhaka Dental College, Dhaka, Bangladesh; ^5^Faculty of Electrical Engineering, FPGA Lab, K. N. Toosi University of Technology, Tehran, Iran; ^6^Omid Hospital, Iran University of Medical Sciences, Tehran, Iran; ^7^Department of Cardiology, National Heart Centre Singapore, Singapore, Singapore; ^8^Duke-NUS Medical School, Singapore; ^9^Harvard Paulson School of Engineering and Applied Sciences, Harvard University, Allston, MA 02134, USA; ^10^Department of Biomedical Engineering, Faculty of Engineering, University Malaya, Kuala Lumpur 50603, Malaysia; ^11^Faculty of Engineering and Built Environment, Universiti Sains Islam Malaysia, Bandar Baru Nilai 71800, Negeri Sembilan, Malaysia; ^12^Department of Biomedical Engineering, Rathinam College of Engineering, Coimbatore, India; ^13^Ngee Ann Polytechnic, Singapore 599489, Singapore; ^14^Department of Biomedical Informatics and Medical Engineering, Asia University, Taichung, Taiwan; ^15^Department of Biomedical Engineering, School of Science and Technology, Singapore University of Social Sciences, Singapore, Singapore

## Abstract

Myocarditis is heart muscle inflammation that is becoming more prevalent these days, especially with the prevalence of COVID-19. Noninvasive imaging cardiac magnetic resonance (CMR) can be used to diagnose myocarditis, but the interpretation is time-consuming and requires expert physicians. Computer-aided diagnostic systems can facilitate the automatic screening of CMR images for triage. This paper presents an automatic model for myocarditis classification based on a deep reinforcement learning approach called as reinforcement learning-based myocarditis diagnosis combined with population-based algorithm (RLMD-PA) that we evaluated using the Z-Alizadeh Sani myocarditis dataset of CMR images prospectively acquired at Omid Hospital, Tehran. This model addresses the imbalanced classification problem inherent to the CMR dataset and formulates the classification problem as a sequential decision-making process. The policy of architecture is based on convolutional neural network (CNN). To implement this model, we first apply the artificial bee colony (ABC) algorithm to obtain initial values for RLMD-PA weights. Next, the agent receives a sample at each step and classifies it. For each classification act, the agent gets a reward from the environment in which the reward of the minority class is greater than the reward of the majority class. Eventually, the agent finds an optimal policy under the guidance of a particular reward function and a helpful learning environment. Experimental results based on standard performance metrics show that RLMD-PA has achieved high accuracy for myocarditis classification, indicating that the proposed model is suitable for myocarditis diagnosis.

## 1. Introduction

Myocarditis is a condition that causes inflammation of the heart muscle [1]. It can affect heart pump function as well as electrical activation and conduction, resulting in heart failure and arrhythmia, respectively. The etiology is diverse, including infection (e.g., viral infections such as COVID-19 and parvovirus) [2], systemic inflammatory and autoimmune diseases, and drug reactions. Symptoms of myocarditis include chest pain, fatigue, and shortness of breath [3]. Patients with suspected myocarditis should seek cardiology advice for early diagnosis and treatment. Endomyocardial biopsy, an invasive procedure, is recommended in severe cases to confirm the diagnosis and to guide treatment [4]. Management comprises supportive measures, symptomatic heart failure therapy, antimicrobials for identified infective agents, and immunosuppression for severe inflammation. Early diagnosis and prompt institution of treatment can significantly reduce morbidity and mortality. Noninvasive cardiac imaging with cardiovascular magnetic resonance imaging (MRI) [5] can help clinch the diagnosis. However, MRI requires expert interpretation, which is manually intensive and subject to operator bias. In this regard, automated diagnostic systems can be developed that employ various machine learning and data mining algorithms to solve medical image classification problems efficiently [6]. They can be applied to reporting workflows to screen images automatically, saving physicians time, reducing errors, and enhancing diagnostic accuracy.

Excellent performance of in-depth models has been demonstrated in diverse applications, including natural language processing [7–9], computer vision, and medical image analysis [10, 11]. Deep learning-based algorithms converge with suitable weights to minimize the error between the real and predicted outputs. Typically, deep models use gradient-based algorithms as backpropagation to learn the weights. However, such optimization methods are sensitive to initial weights and may become trapped in local minima [12]. This issue is mainly encountered during classification [13]. Few researchers have shown that population-based meta-heuristic (PBMH) algorithms [14, 15] may help to overcome this problem [16]. Among PBMH algorithms, the ABC algorithm is one of the most effective optimizers [17, 18]. It emulates the behavior of bees in nature and, unlike traditional optimization algorithms, dispenses with the need to calculate gradients, thereby reducing the probability of getting stuck in local optimizations [19].

Classification performance in many machine learning algorithms may be adversely affected by imbalanced classification [20], which occurs when one class contains disproportionately more data than the others [21]. While imbalanced models may still attain reasonable detection rates for majority samples, the performance for minority samples is weak as minority class specimens can be difficult to identify due to their rarity and randomness. Also, misalignment of minority class samples can result in high costs. Methods have been proposed to address the problem at two levels [22]: data level and algorithmic level. In the former [23–25], training data are manipulated to balance the class distribution by oversampling minority class and/or undersampling majority class [26]. For instance, the synthetic minority oversampling technique (SMOTE) generates new samples by linear interpolation between adjoining minority samples [24], whereas NearMiss undersamples majority samples using the nearest neighbor algorithm [25]. Of note, oversampling and undersampling can risk overfitting and loss of worthy information, respectively [27]. At the algorithmic level, the importance of the minority class can be raised using techniques [28–32] that include cost-sensitive learning, ensemble learning, and decision threshold adjustment. In cost-sensitive learning, different incorrect classification costs are attributed to the loss function for the whole class, with a higher cost being allocated to minority class misclassification. Ensemble learning systems train several subclassifications and then apply voting or combination to obtain better results. Threshold adjustment techniques train the classifier in the imbalanced dataset and modify the decision threshold during the test. Deep learning-based methods have also been suggested for imbalanced data classification [33–35]. The authors in Reference [36] introduced a new loss function for deep networks that could capture classification errors from both minority and majority classes. Reference [37] introduces a method that could learn the unique features of an imbalanced dataset while maintaining intercluster and interclass margins.

To the best of our knowledge, only one work [3] based on deep learning models has been proposed for the diagnosis of myocarditis. The authors developed an algorithm for classifying images based on CNN and the k-means algorithm [38], which has the following workflow: after the data preprocessing stage, the images were placed in several clusters, and each cluster was considered a class in which the CNN classified. The algorithm was repeated for different clusters, and all the results were combined for the final decision. The main problem with the method was that it considered the image matrix as a vector in k-means, which resulted in missed pixels around a specific pixel.

This paper presents a method based on the ABC algorithm and reinforcement learning called RLMD-PA that we believe would address the above mentioned problems. The RLMD-PA model poses the classification problem as a guessing game embodied in a sequential decision-making process. At each step, the agent receives an environmental state represented by a training instance and then executes a classification under the direction of a policy. If the agent performs classification perfectly, it will be given a positive reward and, otherwise, a negative one. The minority class is rewarded more than the majority class. The agent's goal is to accumulate as many rewards as possible during the sequential decision-making process to classify the samples as correctly as possible.

The main contributions of this article are as follows: (1) we considered the classification problem of medical images as a sequential decision-making process. We presented a reinforcement learning-based algorithm for imbalanced classification; (2) instead of randomly weighting, we have developed an encoding strategy and calculated the optimal initial value using the ABC algorithm, and (3) this work is based on a new well-annotated MRI dataset acquired from Tehran's Omid Hospital that we have named the Z-Alizadeh Sani myocarditis dataset and made publicly downloadable.

The rest of the article is structured as follows: the second section is a brief overview of the ABC algorithm and its working. The third section introduces the proposed model. The fourth section presents the evaluation criteria, dataset, and analysis of the results. The last section states the conclusions and future works.

## 2. Background

### 2.1. Artificial Bee Colony Algorithm

Artificial bee colony (ABC) introduced by Karaboga and Basturk [39] is one of the most efficient algorithms for optimizing numerical problems. It is straightforward, robust, and population-based [19]. The algorithm emulates the intelligent foraging behavior of bees to arrive at the optimal solution. There is a list of food sources that bees seek out over time to get to the best positions. The algorithm involves three groups of bees: employed bees, onlooker bees, and scout bees. Employed bees discover the positions of food sources, whereas onlooker bees wait in the hive for the nectar from food positions to be sent by employed bees. Onlooker bees use the information to select food source positions. Once an employed bee has exhausted the food source, it becomes a scout bee to search for new positions randomly. The number of employed bees equals the number of unemployed (onlooker and scout) bees. The steps for optimizing an algorithm using the ABC algorithm are as follows:

(1) Initialization: in the first step, an initial population *S* of size *C* is formed from the positions (solutions), as in
  (1) $$\begin{array}{c} s_{i}^{j}=s_{\min}^{j}+\text{rand}\left(0,1\right)\left(s_{\max}^{j}-s_{\min}^{j}\right), \end{array}$$
where *i* represents the *i*-th position, each solution *s*_*i*_ is *D* dimensions, and *D* means the number of parameters that must be optimized. *s*_min_^*j*^ and *s*_max_^*j*^ are the smallest and largest values in *s*^*j*^, respectively.
(2) Employed bee phase: at this point, new solutions are recognized by searching the neighborhood for current potential solutions. To keep the population size constant, the quality of new solutions is evaluated. If it is better than the previous ones, it will be replaced; otherwise, it will remain fixed. This step can be formed as follows:
  (2) $$\begin{array}{c} v_{i}^{j}=s_{i}^{j}+\varphi_{i}^{j}\left(s_{i}^{j}-s_{k}^{j}\right), \end{array}$$
where *k* is a random solution such that *k* ≠ *i*. *φ*_*i*_^*j*^ is a random number picked from the interval [0, 1]. The potentially new solution *v*_*i*_ is obtained by changing only one element of *s*_*i*_.
(3) Onlooker bee phase: for the onlooker bees update, one solution is stochastically elected from the potential solutions, that is, one of the open facility solutions, according to the probability relation *p*_*i*_ anticipated as follows:
  (3) $$\begin{array}{c} p_{i}=\frac{\text{fit}\left(s_{i}\right)}{\sum_{n=1}^{C}\text{fit}\left(s_{i}\right)}. \end{array}$$
The selection process follows the equation provided: the more appropriate a solution is, the higher the chance it will be selected. If the chosen employed bee scores higher than the current onlooker bee's current solution, the current solution replaces the previous one. This process is repeated for all onlooker bees in population *S*.
(4) Scout bee phase: a solution that does not improve its fit after some repetitions can get the algorithm caught up in local optimization [40]. To prevent this, once the solution's fit does not improve after *t* iterations, the algorithm will discard it, and a new solution will be supplied according to equation (2).
(5) Algorithm end condition: although different conditions can be defined for the end of the algorithm, the term termination is repeated in this study, which means that the algorithm ends after MaxItr iterations.

The complete ABC algorithm is given in Algorithm 1.

### 2.2. Reinforcement Learning

Reinforcement learning [41] is an important branch of machine learning that encompasses many domains. Reinforcement learning can achieve relatively good classification results because it can effectively learn the compelling features of noisy data. In Reference [42], the authors defined classification as a sequential decision problem that used several factors to interact with the environment in order to learn an optimal policy function. Due to the complex simulation between the factors and the environment, the run time was inordinately prolonged. The model presented in [43] is a classification based on reinforcement learning provided for noisy text data. The proposed structure comprises of two classifiers: sample selector and relational classifier. The former selects a quality sentence from the noisy data by following the agent, whereas the latter classifier learns acceptable quality performance from clean data and gives a delayed reward to the sample selector for feedback. Finally, the model yields a superior classifier and quality dataset. The authors in Reference [44] proposed a solution for time series data in which the reward function and Markov process are explicitly defined. In various specific applications [45–48], reinforcement learning has been applied to learn the efficient features. These models promote valuable features for the classification, which leads to higher rewards that guide the agent to select more worthy features. To date, limited work has been done on deep learning for the classification of imbalanced data. In Reference [44], an ensemble pruning technique for deciding subclassifiers that adopted reinforcement learning was proposed. However, the model underperformed when the amount of data was increased. This is because it is difficult to choose classifiers when there are too many subclassifications.

## 3. The Proposed Solution

The overall structure of the proposed model is shown in Figure 1. We considered two critical options for classification. In the first step, we formulated a vector that includes all the learnable weights in our model. We assumed an initial value for the weights with ABC and then applied the backpropagation in the rest of the path. As mentioned, another problem that most classifiers suffer from, including ours, is imbalanced data. To address this, we employed reinforcement learning [49]. These concepts are detailed in the following sections.

### 3.1. Pretraining Phase

Weight initialization of deep networks is an essential part of deep models. Sometimes, incorrect initial values can lead to a failure of convergence in the model. The proposed model has a deep network with weights *θ* that need to be optimized. In this section, we present an encoding strategy and fitness function for the ABC algorithm.

### 3.2. Encoding Strategy

In our work, the encoding strategy aims to arrange the CNN and feed-forward weights in a vector that will be considered the position of the bees in the ABC. Setting the specific weights is a challenge. Nevertheless, we have designed an encoding strategy that is as appropriate as possible after a few experiments.  Figure 2 illustrates an example with encoding of a three-layer CNN network with three filters in each layer and a feed-forward network with three hidden layers. Note that all weight matrices in the vector are stored in rows.

### 3.3. Fitness Function

The fitness function is defined as follows to measure the effectiveness of a solution in the ABC algorithm [12]:

(4) $$\begin{array}{c} \text{Fitness}=\frac{1}{1+\sum_{i=1}^{N}{\left(y_{i}-\hat{y_{i}}\right)}^{2}}, \end{array}$$

where *N* is the total number of samples, and *y*_*i*_ and $\hat{y_{i}}$ are the target and predicted labels for *i*-th data, respectively.

## 4. Classification

Due to the difference in the amount of data between our two classes, we face the problem of imbalanced classification. To address this, we used the imbalanced classification Markov decision process (ICMDP) to construct a sequential decision problem. In reinforcement learning, an agent tries to obtain an optimal policy by performing a series of actions in the environment while maximizing its score. In the case of our model, a sample of the dataset is provided to the agent at each time point and classified. The environment then transmits the immediate score to the agent. A positive score corresponds to a correct rating, whereas a wrong rating gives a negative one. By maximizing cumulative rewards, the agent can arrive at the optimal policy. Let *D*={(*x*_1_, *y*_1_), (*x*_2_, *y*_2_), (*x*_3_, *y*_3_),…, (*x*_*N*_, *y*_*N*_)} be the imbalanced set of existing images with *N* samples, where *x*_*i*_ corresponds to the *i*-th image, and *y*_*i*_ is its corresponding label. The following explains the intended settings:

(i) Policy *π*_*θ*_: policy *π* means a mapping function *S*⟶*A*, where *S* and *A* are a set of states and actions, respectively. In other words, every *π*_*θ*_(*s*_*t*_) means performing the action *a*_*t*_ in the state *s*_*t*_. *π*_*θ*_ is acknowledged as the classifier model with weights *θ*.
(ii) State **s**_**t**_: each state *s*_*t*_ is mapped with sample *x*_*t*_ from the dataset *D*. The first data *x*_1_ are deemed the initial state of *s*_1_. For the model not to learn a particular order, the *D* is shuffled in each episode.
(iii) Action **a**_**t**_: action *a*_*t*_ is performed to predict the label *x*_*t*_. Since the offered classification is binary, *a*_*t*_ ∈ {0,1}, zero represents the minority class and one represents the majority class.
(iv) Reward **r**_**t**_: reward considers the performance of an action. An agent with the correct classification gets a positive reward; otherwise, it gets a negative reward. The amount of this bonus should not be the same for both classes. Rewards can significantly improve model performance because the level of reward and action has been carefully calibrated. In this work, the prize is defined for action according to the following equation [27]:
  (5) $$\begin{array}{c} r_{t}\left(s_{t},a_{t},l_{t}\right)=\left\{\begin{array}{c} +1,a_{t}=y_{t}\text{ and }s_{t}\in D_{H},\\ -1,a_{t}\neq y_{t}\text{ and }s_{t}\in D_{H},\\ \lambda ,a_{t}=y_{t}\text{ and }s_{t}\in D_{S},\\ -\lambda ,a_{t}\neq y_{t}\text{ and }s_{t}\in D_{S}. \end{array}\right. \end{array}$$
where *D*_*H*_ and *D*_*S*_ represent the minority and majority classes, that is, healthy and sick, respectively, and *λ* is a value in the interval [0,1]. The reward *λ* is less than 1/−1 as the minority class becomes more critical due to fewer data. In effect, we can ascribe more importance to the minority class in order for it to approximate the majority class. In the results section, we will see the importance of the value *λ*.
(v) Terminal **E**: the training process is completed at several terminal states, which occur in every training episode. An episode is the transition trajectory from an initial state to a final state, namely, {(*s*_1_, *a*_1_, *y*_1_), (*s*_2_, *a*_2_, *y*_2_), (*s*_3_, *a*_3_, *y*_3_),…, (*s*_*t*_, *a*_*t*_, *y*_*t*_)}. In our case, an episode stops when all the training data have been classified or when a sample of the minority class is misclassified.
(vi) Transition probability **P**: the agent goes from state *s*_*t*_ to the next state *s*_*t*+1_ based on the order of the read data. The transition probability is determined as *p*(*s*_*t*+1_*|s*_*t*_, *a*_*t*_).

In ICMDP, the policy function reports the probability of all labels by receiving a sample:

(6) $$\begin{array}{c} \pi \left(a|s\right)=P\left(a_{t}=a|s_{t}=s\right). \end{array}$$

In reinforcement learning, the intention is to maximize the discounted cumulative reward, or in mathematical terms, to attain a high limit for the following expression:

(7) $$\begin{array}{c} g_{t}=\sum_{k=0}^{\infty }\gamma^{k}. \end{array}$$

Equation (7) is termed the return function, which contains all the accumulated return values of the agent searches in space. The discount factor *γ* ∈ (0,1] [50] is the coefficient of the effect of each reward. The function *Q* measures the quality of a state-action combination:

(8) $$\begin{array}{c} Q^{\pi }\left(s,a\right)=E_{\pi }\left[g_{t}|s_{t}=s,a_{t}=a\right]. \end{array}$$

Equation (8) is expanded according to Bellman's formula [51]

(9) $$\begin{array}{c} Q^{\pi }\left(s,a\right)=E_{\pi }\left[r_{t}+\gamma Q^{\pi }\left(s_{t+1},a_{t+1}\right)|s_{t}=s,a_{t}=a\right]. \end{array}$$

By maximizing the function *Q* supported by *π*, more cumulative rewards can be achieved. The optimal policy of *π*^*∗*^ is assessed by considering the function *Q*^*∗*^ as follows:

(10) $$\begin{array}{c} \pi^{*}\left(a|s\right)=\left\{\begin{array}{cc} 1, & a=\arg\max_{a}Q^{*}\left(s,a\right),\\ 0, & \text{else.} \end{array}\right. \end{array}$$

By combining the two equations (9) and (10), the function *Q*^*∗*^ is expressed as follows [27]:

(11) $$\begin{array}{c} Q^{*}\left(s,a\right)=E_{\pi }\left[r_{t}+\gamma \max_{a}Q^{*}\left(s_{t+1},a_{t+1}\right)|s_{t}=s,a_{t}=a\right]. \end{array}$$

In a low-dimensional space state, the function *Q* can be easily solved by a table. However, the table technique is inadequate when space is joined. To solve this problem, *Q*-learning algorithms are used. In these algorithms, the tuple (*s*, *a*, *r*, *s*_0_) received from equation (11) is saved as experience replay memory *M*. The agent gets a mini-batch *B* from *M* and executes the gradient descent on these data according to the following equation:

(12) $$\begin{array}{c} L\left(\theta_{k}\right)=\sum_{\left(s,a,r,s^{\prime }\right)\in B}{\left(y-Q\left(s,a;\theta_{k}\right)\right)}^{2}, \end{array}$$

where *y* is an estimate of the function *Q* expressed as follows [27]:

(13) $$\begin{array}{c} y=\left\{\begin{array}{cc} r, & \text{end}=\text{True},\\ r+\gamma \max_{a^{\prime }}Q\left(s^{\prime },a^{\prime };\theta_{k-1}\right), & \text{else,} \end{array}\right. \end{array}$$

where *s*′ is the following state *s*, and *a*′ is the action performed in *s*′; end means whether the agent makes a wrong classification for the minority class or not. Finally, the policy weights *π* can be updated as follows:

(14) $$\begin{array}{c} \theta =\theta +l\frac{\nabla L\left(\theta_{k}\right)}{\nabla \left(\theta_{k}\right)},\\ \frac{\nabla L\left(\theta_{k}\right)}{\nabla \left(\theta_{k}\right)}=-2\sum_{\left(s,a,r,s^{\prime }\right)\in B}\left(y-Q\left(s,a;\theta_{k}\right)\right)\frac{\nabla Q\left(s,a;\theta_{k}\right)}{\nabla \left(\theta_{k}\right)}. \end{array}$$

In conclusion, the optimal function *Q*^*∗*^ can be achieved by minimizing the loss function presented in equation (12). Notably, the optimal policy of *π*^*∗*^ is taken using *Q*^*∗*^, which is the optimal model for the proposed classifier.

### 4.1. Overall Algorithm

We devised the simulation environment according to the above. The structure of the policy network depends on the complexity and number of training samples. According to the structure of the training samples and the output, the network input equals to the number of data classes, which is equivalent to 2. The general training algorithm of the RLMD-PA model is displayed in Algorithm 2. In this algorithm, the policy weights are first initialized using the ABC algorithm, and then, the agent continues the training process until an optimal policy is reached. Action is based on a greedy policy, which is also evaluated by Algorithm 3. The algorithm is repeated for *E* times, which is taken as 18,000 in this paper. At each step, the policy network weights are stored.

## 5. Empirical Evaluation

### 5.1. Dataset

Cardiac magnetic resonance imaging (CMR) [52] allows for comprehensive anatomical and functional evaluation of the heart as well as detailed tissue characterization [53]. It is the preeminent imaging modality for noninvasive diagnosis myocarditis without biopsy. The Lake Louise criterion (LLC) [54] introduced benchmark criteria for diagnosing myocarditis using CMR [55] based on the presence of myocardial necrosis, edema, and hyperemia. The presence of late gadolinium enhancement confirms myocardial necrotic damage. T2-weighted images uncover areas of interstitial edema, which indicates inflammatory response. T1-weighted images before and after contrast can depict hyperemia in the myocardial tissue. Fulfilling two of three LLC criteria confers 80% accuracy for diagnosing myocarditis [56]. This article presents a model for identifying myocarditis by considering the three LLC criteria.

A one-year CMR research project on myocarditis was conducted from September 2016 at Omid Hospital in Tehran, Iran, where we performed CMR on patients who were clinically suspected to have myocarditis (e.g., chest pain, elevated troponin, negative functional imaging and/or coronary angiographic findings, and suspected viral etiology) and the treating physician assessed that CMR would likely affect clinical management (e.g., ongoing symptoms, ongoing myocardial injury evidenced by persistent ECG abnormalities, and presence of ventricular dysfunction). The protocol had been approved by the local ethics committee. CMR examination was performed on a 1.5-Tesla system [57]. All cases were scanned with body coils in standard supine position. T1-weighted images were acquired in the axial views. Shortly after gadolinium injection, the T1-weighted sequences were repeated. After approximately 10–15 minutes, late gadolinium enhancement [58] sequences were performed in standard left ventricular short- and long-axis views.  Table 1 summarizes the CMR sequence parameters [3].

A total of 586 patients were identified who had positive evidence of myocarditis on the CMR images, which might show one or more areas of disease. A total of 307 healthy subjects were included as controls. We chose eight CMR images from each patient or control subject for the analysis, which were one long-axis image and one short-axis image acquired using each of the following four CMR sequences: late gadolinium enhancement, perfusion, T2-weighted, and steady-state free precession. The final CMR dataset comprises 4,686 and 2,449 samples from sick (i.e., myocarditis) and healthy subjects, respectively.  Figure 3 shows example images obtained from this dataset. It may be noted that in this study, analysis is performed at the image level, and not at the patient level. In other words, prediction is based on a single image regardless of how many images are available for each patient.

Institutional approval was allowed to use the patient datasets in research studies for diagnostic and therapeutic purposes. Approval was granted on the grounds of existing datasets. Informed consent was received from all of the patients in this study. All methods were carried out in accordance with relevant guidelines and regulations. Ethical approval for using these data was obtained from the Tehran Omid Hospital.

### 5.2. Metrics

To evaluate the classification performance of the proposed model, we used six standard performance metrics, namely, accuracy, recall, precision, *F*-measure, specificity, and *G*-means [59], and they are defined as follows:

(15) $$\begin{array}{c} \text{Accuracy}=\frac{\text{TP}+\text{TN}}{\text{TP}+\text{TN}+\text{FP}+\text{FN}},\\ \text{Recall}=\frac{\text{TP}}{\text{TP}+\text{FN}},\\ \text{Precision}=\frac{\text{TP}}{\text{TP}+\text{FP}},\\ \text{F}-\text{measure}=\frac{2\times \text{Recall}\times \text{Precision}}{\text{Recall}+\text{Precision}}\text{,}\\ \text{Specificity}=\frac{\text{TN}}{\text{TN}+\text{FP}}\text{,}\\ \text{G}-\text{means}=\sqrt{\text{Recall}\times \text{Specificity}}\text{,} \end{array}$$

where TP, TN, FN, and FP are true positive, true negative, false negative, and false positive, respectively. The *F*-measure and *G*-means are commonly applied to evaluate imbalanced classification [27], which aligns nicely with our dataset sample distribution and the reason for existing our proposed method. In addition, it is noteworthy that our prediction is per image. In this way, the intelligent myocarditis classification system can effectively screen entire CMR studies and flag individual images for scrutiny by physician readers. For this purpose, low FP and high recall metrics would be desired.

### 5.3. Details of Model

This work used Python and the PyTorch framework. The codes are written in Jupyter notebook. We used five layers of two-dimensional convolution for the CNN network with 128, 64, 32, 16, and 8 filters. The size of the kernel, stride, and padding in each layer are 3, 2, and 1 for both dimensions, respectively. Each convolution layer involves a max-pooling layer with dimensions of 2 × 2. The three fully connected layers have 128, 64, and 32 hidden layers, respectively. To prevent overfitting, dropout with a probability of 0.4 and early stopping are employed. In every experiment, the batch size is set to 64. The images in the dataset are in gray-scale and light intensities of image pixels are mapped to the range [0, 1]. The images in the dataset come in different sizes and are all resized to 100 × 100 for analysis.

### 5.4. Experimental Results

While standard techniques like data augmentation and weighted loss function [60] can sometimes be used to correct the imbalanced data distributions, they are not applicable in all situations. In our experiments, data augmentation and weighted loss function do not enrich our model, which is not unexpected.

We used *k*-fold cross-validation (*k*=5 or 5-CV) in all our implementations. The entire dataset is divided into *k* subsets. *k* − 1 subsets are applied for training and the remaining one *k* for test. This procedure is iterated *k* times until all data subsets are utilized exactly four times for training and once for testing. All parameters are expressed as means, standard deviations, medians, minimums, and maximums. First, we compared our proposed method with the only published work in this field, CNN-KCL [3]. Next, to investigate the contributions of the two distinct components ABC and RL in our model, we compared the performance of a basic model without ABC and RL, that is, CNN + random weight, versus the models CNN + ABC and CNN + RL, which used ABC and RL for training, respectively. The evaluation results of our RLMD-PA model performance as well as the aforementioned comparisons on the Z-Alizadeh Sani myocarditis dataset are presented in Tables 2 and 3. In general, the RLMD-PA model reduces the error by more than 43%. From the means of all the performance metrics, the RLMD-PA model outperforms the CNN-KCL method as well as CNN + random weight, CNN + ABC, and CNN + RL combinations of its components. Both ABC and RL individually improve on the basic CNN network across all assessed performance metrics, which supports the use of combined approaches of initial weight and reinforcement learning. For better visualization, the results are illustrated in Figure 4. In terms of time, the best model was obtained after 100 iterations in 2 hours, while CNN-KCL got the best after 350 iterations in 5 hours.

Standard machine learning classifiers have not been successful in classifying medical images, because they typically assume images as one-dimensional vectors, which cause the neighboring pixels of a specific pixel to be spaced apart. In order to compare with our deep model, we used five algorithms: support vector machine (SVM) [61], k-nearest neighbor [62], naïve Bayes [63], logistic regression [64], and random forests [65] to classify the CMR images of the study dataset. SVM performed the best among these methods but is still inferior to deep models. The results are summarized in Tables 4 and 5, and the mean performance metrics is shown in Figure 5.

### 5.5. Investigation of Other Metaheuristic Algorithms on the Algorithm

The proposed model employs ABC algorithm in conjunction with backpropagation for the initial value. To compare the performance of ABC versus alternative instructors, we employed ABC in our model with five conventional algorithms, namely, gradient descent with momentum backpropagation (GDM) [66], gradient descent with adaptive learning rate backpropagation (GDA) [67], gradient descent with momentum and adaptive learning rate backpropagation (GDMA) [68], one-step secant backpropagation (OSS) [69], and Bayesian regularization backpropagation (BR) [70], and four metaheuristic algorithms, namely, gray wolf optimization (GWO) [71], the Bat algorithm (BA) [72], Cuckoo optimization algorithm (COA) [73], and whale optimization algorithm (WOA) [74]. The population size and number of function evaluations are 100 and 25,000 for all metaheuristic algorithms, respectively. Other parameter settings can be seen in Table 6. The performance metrics of these comparisons are summarized in Tables 7 and 8 and illustrated in Figure 6. In general, metaheuristic algorithms are better than conventional algorithms with the exception of GDMA in terms of accuracy, recall, and F-measure scores. Importantly, the ABC algorithm outperformed all conventional and metaheuristic algorithms to improve the error in the recall and F-measure criteria by more than 25% and 22%, respectively.

### 5.6. Explore the Reward Function

The reward function is a practical device that helps the agent to achieve the goal. In this work, the minority class reward is +1/−1, while the majority is +*λ*/−*λ*. To examine the effect of the value *λ* on the classification model, we test 10 values of *λ* ∈ {0,0.1, 0.2, 0.3, 0.4, 0.5, 0.6, 0.7, 0.8, 0.9, 1} on the model. Details of the results for all the criteria for these experiments are given in Table 9. For better visualization, we have plotted the trends in Figure 7. On examination, for the accuracy criterion, when *λ* takes the values from [0, 0.3], the chart has an ascending trend, and from [0.3, 1] has a descending move` This process is valid for all criteria. If *λ*=0, the importance of the majority class is disregarded, and if *λ*=1, the importance of both classes is the same. Although the minority class is more important to us, the majority class cannot be ignored.

## 6. Conclusion and Future Directions

This article presents a new model for classifying myocarditis images. The proposed model consists of two steps. First, the model weights are initialized using the ABC algorithm. Next, the model is considered an ICMDP problem. The environment assigns a high reward to the minority class and a low reward to the majority class. The algorithm terminates when the agent makes a wrong classification for the minority class, or the number of episodes runs out. We performed several experiments to examine various factors that affect the performance of the proposed model. The designed experiments confirmed that the RLMD-PA model with ABC and RL is an effective classifier for myocarditis images.

In the future, we will try to employ ensemble convolutional neural network (ECNN), as our model to use a set of CNN networks and connect them to yield higher performance. In addition, we can also work with the generative adversarial network (GAN), which is widely used in many applications. It may be worth exploring to employ the developed model for other medical applications such as stroke detection, cancer detection and plaque detection.

## Figures and Tables

**Figure 1:** Overall process of RLMD-PA.

**Figure 2:** Placement of weights in a vector.

**Figure 3:** Typical healthy and myocarditis images obtained from the Z-Alizadeh Sani myocarditis dataset. The yellow lines indicate the location of myocarditis.

**Figure 4:** Performance of deep learning models on the mean.

**Figure 5:** Performance of traditional methods on the mean.

**Figure 6:** Performance of conventional and metaheuristic models on the mean.

**Figure 7:** Graphical view of change in the performance parameters due to variation in *λ*.

**Algorithm 1:** Pseudocode of the ABC algorithm.

**Algorithm 2:** Pseudocode of the RLMD-PA algorithm.

**Algorithm 3:** Pseudocode of Reward function.

**Table 1:** Characteristics of the Z-Alizadeh Sani myocarditis dataset.

Protocols	TE (mm)	TR (mm)	NF	Slice thickness (mm)	Concatenation and slice number	NE	Breath-hold time (s)
CINE_segmented (true FISP) long axis (LAX)	1.15	33.60	15	7	3	1	8
CINE_segmented (true FISP) short axis (SAX)	1.11	31.92	15	7	15	1	8
T2-weighted (TIRM) LAX, precontrast	52	800	Noncine	10	3	1	9
T2-weighted (TIRM) SAX, precontrast	52	800	Noncine	10	5	1	10
T1 relative-weighted TSE (Trigger)-AXIA-dark blood pre- and postcontrast	24	525	Noncine	8	5	1	7
Late-GD enhancement LGE (high-resolution PSIR) SAX and LAX	3.16	666	Noncine	8	1	1	7

TE: time echo, TR: time repetition, NF: number of frames, NE: number of excitations.

**Table 2:** 5-CV classification performances (accuracy, recall, and precision) obtained for automated myocarditis detection using various combinations of deep learning models with the Z-Alizadeh Sani myocarditis dataset.

	Accuracy					Recall					Precision				
Method	Min	Median	Max	Mean	Std.dev.	Min	Median	Max	Mean	Std.dev.	Min	Median	Max	Mean	Std.dev.
CNN-KCL [3]	0.783	0.811	0.846	0.810	0.024	0.732	0.738	0.807	0.751	0.032	0.704	0.752	0.789	0.745	0.032
CNN + random weight	0.755	0.770	0.807	0.772	0.021	0.695	0.713	0.755	0.717	0.213	0.666	0.685	0.737	0.691	0.029
CNN + ABC	0.799	0.803	0.845	0.815	0.020	0.741	0.766	0.814	0.771	0.027	0.726	0.729	0.783	0.746	0.027
CNN + RL	0.821	0.829	0.869	0.840	0.021	0.762	0.798	0.835	0.801	0.028	0.745	0.772	0.819	0.779	0.029
RLMD-PA (CNN + ABC + RL)	0.862	0.884	0.912	0.886	0.020	0.837	0.869	0.879	0.863	0.017	0.804	0.837	0.886	0.840	0.034

**Table 3:** 5-CV classification performances (F-measure, specificity, and G-means) obtained for automated myocarditis detection using various combinations of methods with the Z-Alizadeh Sani myocarditis dataset.

	F-measure					Specificity					G-means				
Method	Min	Median	Max	Mean	Std.dev.	Min	Median	Max	Mean	Std.dev.	Min	Median	Max	Mean	Std.dev.
CNN-KCL [3]	0.718	0.746	0.798	0.748	0.031	0.814	0.852	0.870	0.845	0.022	0.772	0.795	0.838	0.797	0.025
CNN + random weight	0.681	0.702	0.746	0.704	0.026	0.788	0.800	0.838	0.806	0.020	0.742	0.759	0.795	0.760	0.021
CNN + ABC	0.735	0.745	0.798	0.758	0.026	0.826	0.835	0.864	0.842	0.018	0.787	0.795	0.839	0.806	0.021
CNN + RL	0.767	0.777	0.827	0.790	0.026	0.836	0.864	0.889	0.863	0.020	0.811	0.821	0.862	0.831	0.022
RLMD-PA (CNN + ABC + RL)	0.820	0.847	0.882	0.851	0.024	0.877	0.900	0.932	0.901	0.024	0.857	0.879	0.905	0.882	0.019

**Table 4:** 5-CV classification performances (accuracy, recall, and precision) obtained for automated myocarditis detection using various machine learning algorithms with the Z-Alizadeh Sani myocarditis dataset.

	Accuracy					Recall					Precision				
Method	Min	Median	Max	Mean	Std.dev.	Min	Median	Max	Mean	Std.dev.	Min	Median	Max	Mean	Std.dev.
SVM	0.568	0.691	0.754	0.683	0.070	0.674	0.745	0.778	0.737	0.042	0.450	0.565	0.651	0.565	0.074
KNN	0.480	0.614	0.635	0.588	0.064	0.399	0.637	0.683	0.589	0.111	0.337	0.490	0.511	0.460	0.072
Naïve Bayes	0.547	0.632	0.676	0.615	0.051	0.388	0.534	0.713	0.565	0.134	0.395	0.510	0.553	0.484	0.062
Logistic regression	0.627	0.662	0.720	0.661	0.038	0.583	0.658	0.741	0.657	0.057	0.503	0.542	0.603	0.541	0.041
Random forests	0.415	0.550	0.590	0.530	0.070	0.537	0.683	0.711	0.648	0.071	0.329	0.437	0.469	0.420	0.056

**Table 5:** 5-CV classification performance (*F*-measure, specificity, and *G*-means) obtained for automated myocarditis detection using various machine learning algorithms with the Z-Alizadeh Sani myocarditis dataset.

	*F*-measure					Specificity					*G*-means				
Method	Min	Median	Max	Mean	Std.dev.	Min	Median	Max	Mean	Std.dev.	Min	Median	Max	Mean	Std.dev.
SVM	0.540	0.652	0.695	0.639	0.060	0.505	0.662	0.760	0.651	0.093	0.583	0.704	0.752	0.692	0.065
KNN	0.365	0.554	0.585	0.516	0.089	0.528	0.601	0.629	0.587	0.039	0.459	0.619	0.643	0.587	0.075
Naïve Bayes	0.391	0.522	0.623	0.520	0.092	0.610	0.642	0.692	0.645	0.031	0.499	0.608	0.682	0.600	0.072
Logistic regression	0.565	0.571	0.665	0.593	0.042	0.606	0.665	0.716	0.663	0.049	0.631	0.646	0.724	0.659	0.038
Random forests	0.408	0.533	0.559	0.509	0.063	0.342	0.471	0.529	0.459	0.071	0.429	0.567	0.605	0.545	0.071

**Table 6:** Parameter setting for the experiments.

Algorithm	Parameter	Value
ABC	Limit	*n*_*e*_ × dimensionality of problem
	*n*_*o*_	50% of the colony
	*n*_*e*_	50% of the colony
	*n*_*s*_	1
GWO	No parameters	
BAT	Constant for loudness update	0.50
	Constant for an emission rate update	0.50
	Initial pulse emission rate	0.001
COA	Discovery rate of alien solutions	0.25
WOA	B	1

**Table 7:** Results of 5-CV classification performances (accuracy, recall, and precision) obtained for automated myocarditis detection using various conventional and metaheuristic algorithms with the Z-Alizadeh Sani myocarditis dataset.

	Accuracy					Recall					Precision				
Method	Min	Median	Max	Mean	Std.dev.	Min	Median	Max	Mean	Std.dev.	Min	Median	Max	Mean	Std.dev.
CNN + GDM + RL	0.811	0.857	0.868	0.849	0.022	0.784	0.801	0.830	0.806	0.018	0.732	0.806	0.825	0.796	0.038
CNN + GDA + RL	0.817	0.846	0.857	0.840	0.017	0.784	0.812	0.837	0.808	0.022	0.742	0.786	0.828	0.778	0.035
CNN + GDMA + RL	0.829	0.855	0.887	0.854	0.025	0.764	0.816	0.855	0.817	0.037	0.752	0.809	0.849	0.800	0.037
CNN + OSS + RL	0.823	0.849	0.867	0.846	0.016	0.741	0.814	0.837	0.804	0.037	0.778	0.787	0.814	0.791	0.015
CNN + BR + RL	0.826	0.833	0.855	0.837	0.012	0.745	0.796	0.812	0.785	0.027	0.752	0.761	0.850	0.784	0.041
CNN + GWO + RL	0.833	0.848	0.869	0.850	0.016	0.771	0.796	0.842	0.804	0.027	0.769	0.800	0.816	0.797	0.020
CNN + BAT + RL	0.837	0.847	0.865	0.851	0.013	0.778	0.782	0.833	0.796	0.024	0.787	0.805	0.830	0.807	0.016
CNN + COA + RL	0.815	0.843	0.882	0.844	0.028	0.750	0.826	0.856	0.813	0.046	0.748	0.757	0.838	0.781	0.039
CNN + WOA + RL	0.820	0.845	0.847	0.837	0.012	0.750	0.826	0.814	0.789	0.021	0.742	0.783	0.807	0.781	0.024

**Table 8:** Results of 5-CV classification performances (F-measure, specificity, and G-means) obtained for automated myocarditis detection using various conventional and metaheuristic algorithms with the Z-Alizadeh Sani myocarditis dataset.

	*F*-measure					Specificity					*G*-means				
Method	Min	Median	Max	Mean	Std.dev.	Min	Median	Max	Mean	Std.dev.	Min	Median	Max	Mean	Std.dev.
CNN + GDM + RL	0.757	0.811	0.825	0.801	0.026	0.827	0.882	0.898	0.875	0.028	0.805	0.848	0.860	0.840	0.021
CNN + GDA + RL	0.765	0.799	0.811	0.792	0.019	0.834	0.863	0.902	0.860	0.028	0.812	0.839	0.850	0.834	0.015
CNN + GDMA + RL	0.771	0.806	0.849	0.808	0.033	0.838	0.880	0.909	0.877	0.026	0.815	0.843	0.878	0.846	0.026
CNN + OSS + RL	0.759	0.799	0.825	0.797	0.024	0.859	0.873	0.885	0.872	0.010	0.804	0.839	0.861	0.837	0.021
CNN + BR + RL	0.776	0.784	0.794	0.784	0.007	0.841	0.850	0.921	0.868	0.034	0.821	0.825	0.829	0.825	0.003
CNN + GWO + RL	0.779	0.797	0.828	0.801	0.021	0.856	0.880	0.889	0.877	0.013	0.821	0.836	0.863	0.840	0.018
CNN + BAT + RL	0.782	0.793	0.823	0.801	0.018	0.873	0.885	0.901	0.885	0.010	0.824	0.832	0.859	0.839	0.016
CNN + COA + RL	0.752	0.803	0.844	0.796	0.038	0.835	0.854	0.901	0.862	0.028	0.800	0.845	0.876	0.837	0.031
CNN + WOA + RL	0.768	0.793	0.798	0.785	0.014	0.832	0.869	0.888	0.866	0.021	0.812	0.832	0.839	0.827	0.012

**Table 9:** Performance evaluation obtained for various values of *λ* as the reward of the majority class.

*λ*	Accuracy	Recall	Precision	*F*-measure	Specificity	*G*-means
0	0.807	0.778	0.727	0.752	0.824	0.801
0.1	0.838	0.814	0.769	0.791	0.853	0.833
0.2	0.867	0.844	0.810	0.827	0.880	0.862
0.3	0.884	0.858	0.837	0.847	0.900	0.879
0.4	0.877	0.848	0.830	0.839	0.895	0.871
0.5	0.857	0.814	0.807	0.810	0.883	0.848
0.6	0.845	0.798	0.792	0.795	0.874	0.835
0.7	0.825	0.764	0.768	0.766	0.861	0.811
0.8	0.807	0.738	0.746	0.742	0.848	0.791
0.9	0.792	0.709	0.730	0.719	0.842	0.773
1	0.779	0.695	0.710	0.702	0.829	0.759

## Data Availability

The dataset used to support the findings of this study is available on GitHub: https://github.com/vahid-moravvej/Z-Alizadeh-Sani-myocarditis-dataset.
